The article "A Case Report of Grisel’s Syndrome Complicating the Postoperative Course of Craniotomy for a Massive Cystic Brain Lesion" was retracted in 2025. Reason: concerns about the authorship.

# A Case Report of Grisel’s Syndrome Complicating the Postoperative Course of Craniotomy for a Massive Cystic Brain Lesion

**DOI:** 10.7759/cureus.73776

**Published:** 2024-11-15

**Authors:** Takara R Newsome-Cuby, Kwadwo Darko, Peace Odiase, Sean O'Leary, Charles Marchese, Michael J Valentine, Benjamin Pautler, Usama AlDallal, Mohamed Ismail, Fakhar Hayat

**Affiliations:** 1 School of Osteopathic Medicine, Kansas City University, Kansas City, USA; 2 Neurosurgery, Korle-Bu Teaching Hospital, Accra, GHA; 3 Biochemistry and Cancer Biology, Meherry Medical College, Nashville, USA; 4 Neurosurgery, University of Texas Medical Branch at Galveston, Galveston, USA; 5 School of Medicine, Royal College of Surgeons In Ireland - Medical University of Bahrain, Busaiteen, BHR; 6 Neurosurgery, King Hamad University Hospital, Busaiteen, BHR

**Keywords:** atlantoaxial rotatory subluxation, brain lesion, decompressive craniotomy, grisel’s syndrome, halo vest, neurological symptoms in pediatric age group

## Abstract

This report presents the case of a seven-year-old child diagnosed with Grisel’s syndrome following a craniotomy for a cystic brain lesion. The patient initially presented with persistent, progressively worsening headaches that coincided with neurological symptoms. Imaging revealed a massive cystic lesion causing a significant compression and midline shift. Following craniotomy and insertion of a left frontal Ommaya reservoir, the patient developed Grisel’s syndrome, characterized by painful neck muscle spasms and rotation to the right. Management included the application of halo traction to ensure rigid cervical spine immobilization, closed reduction, and subsequent transition to a halo vest to maintain alignment and facilitate gradual recovery.

## Introduction

Grisel’s syndrome, a rare yet clinically significant condition, is characterized by non-traumatic subluxation of the atlantoaxial joint, often associated with inflammatory processes in the head and neck. This syndrome typically arises following inflammatory conditions affecting the upper neck or otolaryngological surgical procedures [1]. It is commonly observed in children as acute torticollis and atlantoaxial joint subluxation secondary to inflammation [2].

The pathophysiology of Grisel’s syndrome is believed to involve the spread of infection up the cervical vertebrae, leading to laxity of the atlantoaxial ligament complex and subsequent subluxation of the atlantoaxial joint [3,4]. Given the severity of complications that may arise in the mastoid, throat, and air sinuses, timely recognition and appropriate treatment are critical for effectively mitigating these risks. Grisel’s syndrome is also associated with sinusitis and other inflammatory conditions of the adjacent neck tissues [5]. Furthermore, this syndrome predominantly affects children, adding to the importance of accurate diagnosis and the urgency of its management [6]. Hence, understanding its pathophysiology, risk factors, clinical presentation, and management strategies is crucial.

In this case report, we discuss a seven-year-old female patient who presented with recurrent headaches, seizures, and ataxia. Subsequently, she developed Grisel’s syndrome post-craniotomy. This report aims to contribute to the current literature on Grisel's syndrome.

## Case presentation

Patient presentation

A seven-year-old female patient presented with multiple headaches of approximately a year's duration. Over four weeks, her headaches increased in their severity. Initially, her symptoms included weekly headaches accompanied by vomiting. However, their frequency increased to every three to four days and was associated with instability, an inability to walk, episodic nausea, and recurrent fever. There was no loss of consciousness or vision changes, but she did exhibit single jerk movements of the limbs and trunk upon presentation. Notably, developmental delays were also present, including speech delay, learning difficulties, and memory problems. There was no known family history of similar conditions.

Clinical findings and diagnostic assessment

Clinically, the patient was conscious with a Glasgow Coma Scale score of 15/15 and presented with a low-grade fever. Neurological examinations revealed spastic lower limbs, right hemiplegia, a positive Romberg's sign, and bilateral Babinski sign with intact cranial nerves and cerebellar function. An ophthalmological review showed Grade 2 papilledema with a normal macula and peripheries. Computed tomography (CT) brain (Figures 1A, 1B) identified a large cystic lesion in the left fronto-temporo-parietal region, causing compression of the left lateral ventricle, a midline shift, and compression of the third ventricle with mild-to-moderate hydrocephalus and transependymal edema. Together, these images suggested a neuroglial cyst, a cystic tumor, or a parasitic cyst.

**Figure 1:** Computed tomography (CT) brain A. Sagittal view showing a large fronto-temporo-parietal intra-axial cystic lesion (red arrow) measuring 12 x 8.6 x 9.5 cm with a thin wall, focal calcifications, and mild edema B. Axial cut showing the cystic lesion (red arrow) causing significant mass effect with a 17.5 mm midline shift to the right, compression of the left lateral and third ventricles, resulting in mild-to-moderate dilatation of the ventricular system and transependymal edema.

Differential diagnoses included low-grade tumors such as desmoplastic infantile ganglioglioma and high-grade tumors like primitive neuroectodermal tumors. The imaging also revealed obstructive hydrocephalus with CSF seepage and contralateral acute hydrocephalus. Her treatment regimen included phenytoin (50 mg thrice daily), dexamethasone (2mg thrice daily), omeprazole (40 mg IV), and paracetamol (420 mg thrice daily).

Course of admission

The patient was admitted and commenced on a regimen including ibuprofen (250 mg oral syrup every eight hours as needed), dexamethasone (2 mg IV every eight hours), ceftazidime (1,500 mg IV three times daily), levetiracetam (500 mg IV twice daily), and omeprazole (20 mg once daily). Preparations were made for an urgent left fronto-temporo-parietal craniotomy to perform an excisional biopsy. During the surgery, a massive cystic lesion was discovered in the left frontal lobe, exerting pressure on the brain stem. The patient underwent the insertion of a left frontal Ommaya reservoir and was then transferred to the pediatric intensive care unit (PICU). There, she was ventilated and successfully extubated the following day.

She was then moved to the general ward for continued medical management and physiotherapy rehabilitation. Seven weeks into her admission, she developed neck muscle spasms, resulting in rightward rotation and painful movement limitations. A CT (Figures 2A, 2B) and magnetic resonance imaging (MRI) (Figures 3A, 3B) of the cervical spine were conducted, leading to a diagnosis of torticollis secondary to Grisel's syndrome.

**Figure 2:** Computed tomography (CT) cervical A. 3D-CT reconstruction image, showing rightward atlanto-axial rotation (red arrow). B. Plain CT of the C-spine showing asymmetrical lateral atlantodental joint spaces with widened left side measured 6.5 mm and anticlockwise rotation C1 on C2 (red arrow).

**Figure 3:** MRI sagittal T2 sequence A. 3D-CT reconstruction image showing reduction in the asymmetry of the lateral atlantodental joint spaces and realignment of the C1 vertebra on the C2 vertebra (red arrow). B. Plain CT of the cervical spine demonstrating symmetric lateral atlantodental joint spaces. The previously noted anterior subluxation of the right occipital condyle relative to the right lateral mass of the C1 vertebra, observed in prior imaging, is no longer evident.

Management included avoiding head rotation and aggressive neck movements, using a soft neck collar, continuing active physiotherapy thrice daily, and applying Voltaren gel on the neck.

Discharge and follow up

After the patient was diagnosed with Grisel's syndrome, a halo traction device was placed for stabilization, leading to an improvement in the patient’s symptoms. She was eventually discharged and followed up at the neurosurgery outpatient department. 

Approximately two months after the halo vest was applied, the patient returned with head pain caused by a displaced left frontal screw on the crown component of the halo fixation system, which was subsequently repositioned. After four months, the halo vest was removed under sedation, and a Miami J hard neck collar (Jerome Medical, Moorestown, NJ) was applied. She wore the Miami J collar for two months, after which serial cervical X-rays and CT scans were conducted. Following these assessments, she transitioned to a soft cervical collar for gradual weaning off neck support.

At her last follow-up at eight months, she reported no seizures, despite poor adherence to the dosing schedule of her anti-seizure medications. Her parents expressed concerns about her poor concentration, declining school performance, and occasional emotional outbursts.

## Discussion

Grisel's syndrome is an uncommon condition characterized by rotational atlantoaxial subluxation without the presence of trauma. The majority of cases are observed in the pediatric demographic, with 68% occurring in children younger than 12 years old and 90% under the age of 21 [7,8]. Persistent torticollis and nuchal muscle spasms are common indicators for diagnosing Grisel's syndrome. Surgical intervention in the head and neck regions and/or upper respiratory tract infections emerge as the most frequently reported triggers [8]. CT of the neck is the preferred diagnostic method for revealing atlantoaxial subluxation and rotation. In addition, MRI can reveal inflammatory changes in the adjacent soft tissues and provide resolution for alterations in the alar and transverse ligaments, and possible spinal cord compression [9].

The brain lesion in this patient was characterized by reactive gliosis, with features suggestive of pilocytic astrocytoma. The exact pathogenesis of Grisel's syndrome in this context remains elusive but may involve neuromuscular injury, considering the patient's postoperative course. Atlantoaxial subluxation in Grisel's syndrome is attributed to increased laxity of the joint ligaments caused by localized hyperemia and inflammatory response due to infections or surgical intervention [10]. In our case, post-surgical trauma resulted in localized inflammation leading to the diagnosis of this syndrome [11]. In adults, the typical atlas-dens interval ranges from 2.5 to 3 mm, whereas in children, this interval expands to 4.5 mm [12]. This inherent cervical ligamentous laxity in the stabilizing soft tissues of C1 and C2 is commonly observed in the baseline pediatric population and increases the chances for atlantoaxial subluxation in children.

Grisel's syndrome is a rare but serious condition, particularly when it complicates postoperative care. Its occurrence following neurosurgical intervention, as observed in this case, underscores the need for vigilant monitoring for potential cervical instability. Conservative treatment, such as halo fixation or cervical collars, has been shown to improve cervical alignment without the need for surgery. Like in this case, a meta-analysis of 119 cases showed that 93% of post-surgical patients were managed successfully with conservative treatment [13].

Continued correlation with imaging, such as MRI, is advised to further evaluate the brain lesion and definitively rule out pilocytic astrocytoma. Long-term follow-up should encompass neurological assessments and imaging studies to monitor the resolution or progression of the brain lesion and potential recurrence of Grisel's syndrome. Overall, we recommend that this syndrome be considered for observation - especially after invasive procedures are performed near the craniovertebral junction in the pediatric population.

## Conclusions

This case illustrates the rare occurrence of Grisel's syndrome, complicating the postoperative course of a child following craniotomy for a massive cystic brain lesion. Vigilant monitoring, prompt diagnosis, and appropriate intervention, including traction and halo vest application, were crucial in managing this complex condition. Long-term follow-up and multidisciplinary care remain essential for optimal patient outcomes.
